# The Supervision Mechanism of Residents' Waste Separation Behavior: Analysis Using a Tripartite Evolutionary Game Model

**DOI:** 10.1155/2023/2551973

**Published:** 2023-01-31

**Authors:** Mengge Hao, Shichun Xu, Jingnan Zhang, Xiaona Meng

**Affiliations:** School of Economics and Management, China University of Mining and Technology, Xuzhou 221116, China

## Abstract

To promote residents' waste separation behavior, waste separation supervision has been a crucial need. This paper aims to explore the supervision mechanism of residents' waste separation behavior using a tripartite evolutionary game model. The evolutionary stability conditions of resident, property service enterprise, and the government were analyzed. The influences of the main parameters on the strategy of three stakeholders were explored through numerical simulation. The results show that the regulatory mechanism of waste separation will reach the optimal stable strategy when the following conditions are satisfied: (1) the penalty for nonclassification is higher than the difference between classification cost and the total benefit of classification; (2) the subsidy to property services enterprise is greater than the total cost of positive participation management. Residents' behaviors are mainly influenced by rewards and punishments. The behavioral strategies of property service companies are more sensitive to subsidies than penalties. In the early stage of mandatory waste separation, it is important to reduce the cost of residents' separation, develop the publics' environmental awareness, and increase the willingness of properties to participate in management. This paper presents a new perspective and theoretical guidelines for the local government and communities to supervise residents' waste separation behaviors in China and other developing countries and offers useful insights into waste separation management for other countries.

## 1. Introduction

According to the World Bank, global municipal waste generation will reach 3.4 billion metric tons by 2050. The enormous amount of municipal solid waste generated and improper disposal will consume huge resources and seriously threaten the ecological environment. Waste separation is widely recognized as an effective way to reduce municipal solid waste generation and increase resource utilization [1, 2]. Countries around the world are actively promoting waste separation, so as to resolve the environmental problems caused by municipal solid waste. Most developed countries have implemented sound waste management regulations and established waste separation systems [3]. The United States has adopted new regulations to guide local governments to provide recycling services to households and implement curbside pricing programs [4]. Japan has made remarkable achievements in waste separation, recovering a variety of resources from solid waste each year. The mature waste disposal industry has been established in Germany, providing employment for 25 million people and accounting for 1.5% of the national economy in terms of turnover [5]. However, many developing countries, such as China, Brazil, India, Ghana, and Palestine, face enormous challenges in guiding residents to separate their waste, including poor public attitude, inadequate regulation, and insufficient infrastructure [6–8]. In Abaqulusi, South Africa, only 16% of households participated in waste separation practices [9]. Meanwhile, some measures employed by some developed countries, such as pay-as-you-throw, which is not yet appropriate for developing countries due to their underdeveloped economies [10]. Thus, it is necessary to study waste separation in developing countries to explore sustainable solid waste management suitable for these countries.

China, as one of the largest developing countries, has introduced many measures to guide residents to participate in waste separation. The State Council of China suggested in 2016 that the establishment of a coordination mechanism between the government, communities, enterprises, and residents could promote waste reduction and separation. The local governments actively respond to the central government's instructions and issue mandatory waste separation policies [11]. Many measures to guide residents to sort waste at source are characterized by penalties and incentives. For example, 50–200 yuan (about US$7.91–31.66) would be fined for residents refusing to separate waste in Shanghai. Residents with outstanding achievements in waste sorting would be rewarded. Domestic waste management in residential communities is one of the property service companies' daily routines in China. The mandatory policy states that the property service enterprise is responsible for waste separation management in the community, including providing waste separation infrastructure, instructing residents to sort waste, and stopping nonseparation behavior. The property service enterprises who fail to manage the waste separation as required would be fined 500–5000 yuan (about US$79.15–791.50). Although the mandatory waste separation policy offers new ideas for solid waste management in developing countries, there are still some dilemmas. For example, the participation rate in waste separation is low [12], and the residents have not formed the habit of waste separation [13]. The reasons for these dilemmas include inadequate supervision and poor coordination among departments [14]. Thus, it is important to explore the waste separation supervision mechanism in order to encourage the collaborative participation of departments. Considering the specific institutional environment brought by the mandatory waste separation policy and the fact that China is in the stage of economic transition, it would be helpful for China and other developing countries' solid waste management and sustainability to explore the supervision mechanism for residents' waste separation behavior.

The evolutionary game theory, unlike the classical traditional game theory, supposes that the participants are finitely rational and focuses on the dynamic process of a stable state and the specific change of the system [15]. Each stakeholder in solid waste management has bounded rationality and adopts different behavioral decisions depending on changes in revenues and costs. Although some studies have investigated solid waste management using evolutionary games, research on the supervision mechanism of waste separation is rare, especially in the context of China's mandatory waste separation policy. There may be a direct link between the strength of regulation and the effectiveness of the mandatory policy, as most residents are less likely to participate in waste separation without supervision [16, 17]. The evolutionary game model can explain the dynamic interactions of stakeholders under the mandatory policy and try to solve the dilemma of waste separation governance. Therefore, it is a reasonable choice to systematically reveal the behavioral decision-making in the process of waste separation supervision in China using evolutionary game theory. In addition, the existing related literature mainly discusses the game relationship between recycling companies and government, as well as between residents and government, ignoring the role of property service companies in waste separation supervision. China's new waste separation policy stipulates that residents must dump their garbage in specific bins at scheduled times in the presence of a supervisor [4], indicating that property service companies have to take on the supervision of residential communities. In this regard, property service enterprises are introduced into the evolutionary game model to analyze the behavioral strategies of residents, property service enterprises, and the government in the waste separation supervision system. Furthermore, the effects of the main parameters on the waste separation regulatory system were analyzed. On the theoretical side, this study makes a meaningful contribution to the literature by introducing property service companies into the regulatory model of residents' waste separation behavior. On the practical side, our study could provide a practical reference for waste separation management in China and other developing countries.

The remaining parts of this paper are designed in the following manner: Section 2 reviews the existing studies.  Section 3 presents the model construction and solution. The simulation analysis is revealed in Section 4. The discussion of the mina results is shown in Section 5.  Section 6 puts forward conclusions and policy recommendations for improving residents' waste separation behavior.

## 2. Literature Review

The initial research on solid waste focused on generation forecasting and solid waste management assessment. For example, Al-Subu et al. [18] predicted the amount and components of municipal solid waste in Nablus and Jenin Districts, West Bank, using regression predictive models. Al-Khateeb et al. [19] and Al-Batnij et al. [20] assessed solid waste management in Palestine.

Given the importance of waste separation for environmental sustainability, residents' waste sorting behavior and its influencing factors were investigated [21]. Most studies suggest that psychological factors (such as environmental cognition, sense of social responsibility, attitude, personal norms, perceived behavioral control, and willingness to waste separation) positively affect waste sorting behavior [22–29]. Oehman et al. [30] found that attitudes, subjective norms, and perceived behavioral control were positively associated with willingness to separate household food waste. Al-Subu et al. [31] studied residents' concerns and attitudes towards the implementation of solid waste management facilities in the Nablus and Jenin Districts of Palestine. Situational factors (such as time, space, infrastructure, and policy measures) are closely related to the convenience and cost of waste separation and significantly positively affect residents' waste separation behavior [32, 33]. For instance, Cheng et al. [34] found that about 85% of the residents would sort their waste when the perceived convenience of infrastructure was high. Based on the cost uncertainty, Ma et al. [35] proposed an incentive strategy model to improve the public awareness of waste sorting.

Many studies explored how to motivate people to engage in waste separation practices [23, 36]. The effect of different information interventions on the recurrence of residents' waste sorting behavior was investigated by Chen et al. [37]. The penalty and reward were considered effective measures [38]. Asare et al. [39] indicated that the rewards increased the waste separation efficiency and recycling rate of recyclable waste in Ghana. Many studies, such as Struk [40], Abila and Kantola [41], and Alhassan et al. [42], pointed out that economic incentives can improve municipal waste management and reduce the amount of waste generated in Ghana, Finland, and Italy. Chen et al. [43] found that the proportion of residents' positive emotion toward mandatory waste separation policy showed a trend of decreasing first and then increasing. The penalties have some side effects [44, 45], and most studies suggest that the rewards are more effective than penalties in promoting peoples' waste sorting behavior [2]. However, the government prefers to conduct penalty measures because it facilitates large-scale administration and creates financial interest for the government [2]. Therefore, it is still worth studying the incentive measures to mobilize residents to participate in waste separation.

Waste management is characterized by public products, nonexclusive and noncompetitive from the economic perspective, so public tragedy and prisoners' dilemmas occur [46, 47]. Many studies applied the evolutionary game theory to analyze stakeholders' behavior in the area of solid waste management, such as construction and demolition waste [48–50], industrial waste [51], e-waste [52], food waste [53, 54], plastic waste [55], and express packaging waste [56]. Some scholars studied the behavioral decisions of stakeholders in the process of waste separation and recycling. For example, Chen et al. [47] constructed a reticular cooperative waste sorting mode involving an individual and another individual to analyze the residents' behavioral strategy choice in the situations of independent separation and cooperative separation. Zhang [57] compared the static and dynamic penalty mechanisms for waste separation to analyze the behavioral strategies of the public and the government. Wu et al. [17] established the evolutionary game model involving the government and residents in municipal household waste separation. Based on the prospect theory and evolutionary game, Zhang et al. [58] investigated the behavior change process of government and residents to understand how to optimize the benefits of waste separation for stakeholders. Chen and Gao [59] analyzed the behavioral strategies of residents, waste disposal companies, and the government in waste separation and recycling using evolutionary games and studied the stability of the evolutionary system through multi-agent-based simulation. Teng et al. [60] investigated the behavioral decision-making of village collectives in rural waste classification by constructing a tripartite evolutionary game model involving farmers, village collectives, and the government.

The existing studies mainly present the following shortcomings: First, most previous studies focus on the waste recycling formed by the waste disposal enterprises, waste recycling enterprises, the government, and others, but few research explores the characteristics and rules of residents' waste separation behavior and the supervision mechanism under the mandatory waste separation policy in China. The residents' behaviors, as the source of waste separation activity, have an important impact on the waste separation management system, so the residents' waste separation behavior should be the main research subject. Second, most studies related to waste separation only concern the interactions between two stakeholders (such as residents and the government) and ignore the crucial role of supervision at the community level. In reality, it is difficult for the government to directly supervise the public's behavior [5], so the property service enterprises' participation in waste separation management at the community level should be valued.

With respect to existing literature, this study analyzes the behavioral strategies of the three participants in the waste separation supervision system. A tripartite evolutionary game model is first structured, and then the evolutionary stability strategy (ESS) is derived by solving the replicator dynamic equations of the three participants. According to the Lyapunov stability method, the stability conditions of equilibrium points are obtained. The validity of the supervision mechanism for waste separation is further verified through numerical simulation. The main contributions of this study are emphasized below. First, we proposed a tripartite evolutionary game model consisting of residents, property service enterprises, and the government. Different from previous studies, the tripartite evolutionary game model constructed in this paper is consistent with the reality of waste separation management in China under the mandatory policy and explains the role of property service companies in the third-party supervision of waste separation. Second, the impacts of main factors, such as intention, reward, subsidy and penalty, on the evolution to the optimal stability strategy, are explored through numerical simulation, so as to explore incentives measures to promote residents' participation in waste separation.

## 3. Evolutionary Game Model

### 3.1. Model Description and Assumption

Residents, property service enterprises, and government are the main participants in the waste separation supervision system in China. They can choose a certain strategy due to the changes in benefits and costs. The following game strategies of the three stakeholders in the system are expressed.

The resident' behavioral choices are divided into classification behavior and non-classification behavior. The classification behavior means that residents separate their waste at source according to the requirements specified in the mandatory policy. The non-classification behavior represents that the resident does not separate waste as required.

The property service enterprise has two behavioral choices, namely, positive participation management and negative participation management. Positive participation management means that the property service enterprise update and maintain waste separation infrastructures such as smart waste bins in the community, the instructor equipped to guide residents to separate waste, and persuasion for residents who do not separate waste. The negative participation management means that property service enterprise continues to use traditional garbage cans and does not employ supervisors to guide residents to sort waste.

The government is the regulator of irregularities that has two behavioral choices, namely, strict supervision and loose supervision. If the government chooses the strategy of strict supervision, violations by property service enterprises are bound to be detected by the government. Under loose supervision, the government has a certain probability to find the illegal behavior of property service enterprises.

The following assumptions are proposed based on the dynamic game relationships among the three participants:

1. The resident, property service enterprise, and government are bounded with rationality.
2. We suppose that the probability that residents adopt classification behavior is *x*, and the probability of adopting non-classification behavior is 1 − *x*. The probability that the property service enterprise adopts positive participation management is *y*, and the probability of adopting negative participation management is 1 − *y*. The probability that the government adopts strict supervision is *z*, and the probability of adopting loose supervision is 1 − *z*.
3. The resident with classification behavior will take time to learn the knowledge and methods of waste separation and sort their waste as required in daily life. Their cost of adapting classification behavior is *C*_1_, and they can gain the revenue *R*_1_ (such as the sanitary and beautiful living environment). If residents choose classification behavior, the property service enterprise gets the benefits *R*_2_ (such as improved resource utilization and reputation). The waste separation will produce environmental and social benefits *R*_3_ owned by the government, because it contributes to the improvement of the ecological environment.
4. If the property service enterprise chooses positive participation management, the investment cost in human resources, material resources, and financial resources is denoted by *C*_2_. In the management process, the property service enterprise will reward the residents who choose classification behavior *H*_1_ (such as green points and gifts) and punish the residents who do not separate waste *f*_1_ (such as fines and voluntary labor).
5. As a regulator, the government inspects whether the property service enterprise's actions comply with the requirements of the mandatory policy. The government with the behavior strategy of strict supervision will need to invest additional human, material, and financial costs denoted by *C*_3_. The government provides subsidy *H*_2_ to the property service enterprises that choose the behavioral choices of positive participation management.
6. When the resident chooses classification behavior and the property service enterprise chooses negative participation management, the waste will be classified. When the resident chooses non-classification behavior and the property service enterprise chooses to actively participate in the management, the instructor will require the residents who failed to sort their waste to correctly place waste. Thus, in the two cases, the government will get environmental and social benefits *R*_3_. If and only if residents do not sort waste and the property service enterprises negatively participate in the management at the same time, there will be violations of mixed waste collection and transportation. The government choosing strict regulation will detect violations, while those who choose loose regulation have a probability of finding irregularities (the probability is *a*). Thus, the government imposes the penalty *f*_2_ for the property service enterprise choosing negatively participation. In addition, the government pays extra treatment costs for unclassified waste pollution, and the treatment cost is represented by *C*_4_. All the parameters are positive, and *x*, *y*, *z* ∈ [0,1], 0 < *a* < 1.

Based on the previous assumptions, the tripartite game tree of residents, property service enterprises, and the government is shown in Figure 1.

### 3.2. The Payoff Matrix and Game Equilibrium Point

Table 1 shows the payoff matrix for the three stakeholders. According to Table 1, the expected benefit functions of residents adopting classification behavior and non-classification behavior can be obtained and expressed as *E*_*x*_, *E*_1−*x*_, respectively. This can be shown as equations (1) and (2).

(1) $$\begin{array}{c} E_{x}=z\left[y\left(R_{1}+H_{1}-C_{1}\right)+\left(1-y\right)\left(R_{1}-C_{1}\right)\right]+\left(1-z\right)\left[y\left(R_{1}+H_{1}-C_{1}\right)+\left(1-y\right)\left(R_{1}-C_{1}\right)\right]=yH_{1}+R_{1}-C_{1}\text{,} \end{array}$$

(2) $$\begin{array}{c} E_{1-x}=z\left[y\left(-f_{1}\right)+\left(1-y\right)\left(0\right)\right]+\left(1-z\right)\left[y\left(-f_{1}\right)+\left(1-y\right)\left(0\right)\right]=-yf_{1}\text{.} \end{array}$$

The replicator dynamic equation of resident adopting classification behavior is expressed in equation (3).

(3) $$\begin{array}{c} F\left(x\right)=\frac{dx}{dt}=x\left(1-x\right)\left(E_{x}-E_{1-x}\right)=x\left(1-x\right)\left[y\left(H_{1}+f_{1}\right)+R_{1}-C_{1}\right]\text{.} \end{array}$$

We use *E*_*y*_ and *E*_1−*y*_ to denote the expected benefit functions of property service enterprise adopting positive participation management and negative participation management, respectively. The replicator dynamic equation of property service enterprise adopting positive participation management is expressed in equation (4).

(4) $$\begin{array}{c} F\left(y\right)=\frac{dy}{dt}=y\left(1-y\right)\left(E_{y}-E_{1-y}\right)=y\left(1-y\right)\left[-xz\left(1-a\right)f_{2}-x\left(H_{1}+f_{1}+af_{2}\right)+z\left(1-a\right)f_{2}+f_{1}+H_{2}-C_{2}+af_{2}\right]\text{.} \end{array}$$

Similarly, we denote the expected benefit functions of the government adopting strict supervision and loose supervision by *E*_*z*_ and *E*_1−*Z*_, respectively. The replicator dynamic equation of the government adopting strict supervision is expressed in equation (5).

(5) $$\begin{array}{c} F\left(z\right)=\frac{dz}{dt}=z\left(1-z\right)\left(E_{z}-E_{1-Z}\right)=z\left(1-z\right)\left[xy{\left(1-a\right)f}_{2}-x\left(1-a\right)f_{2}-y\left(1-a\right)f_{2}+{\left(1-a\right)f}_{2}-C_{3}\right]\text{.} \end{array}$$

### 3.3. The Solution of Evolutionary Stability Strategy

The waste separation supervision system based on the evolutionary game theory is composed of equations (3)–(5). This can be represented in equation (6).

(6) $$\begin{array}{c} \left\{\begin{array}{l} F\left(x\right)=x\left(1-x\right)\left[y\left(H_{1}+f_{1}\right)+R_{1}-C_{1}\right]\text{,}\\ F\left(y\right)=y\left(1-y\right)\left[-xz\left(1-a\right)f_{2}-x\left(H_{1}+f_{1}+af_{2}\right)+z\left(1-a\right)f_{2}+f_{1}+H_{2}-C_{2}+af_{2}\right]\text{,}\\ F\left(z\right)=z\left(1-z\right)\left[xy\left(1-a\right)f_{2}-x\left(1-a\right)f_{2}-y\left(1-a\right)f_{2}+{\left(1-a\right)f}_{2}-C_{3}\right]\text{.} \end{array}\right. \end{array}$$

Let three replicator dynamic equation be equal to 0, that is, *F*(*x*)=0, *F*(*y*)=0, *F*(*z*)=0. This study derives eight pure strategy equilibrium points, i.e., *E*_1_(0, 0, 0), *E*_2_(0, 0, 1), *E*_3_(0, 1, 0), *E*_4_(0, 1, 1), *E*_5_(1, 0, 0), *E*_6_(1, 0, 1), *E*_7_(1, 1, 0), and *E*_8_(1, 1, 1). At the same time, there exists a mixed strategy solution *E*_9_(*x*^*∗*^, *y*^*∗*^, *z*^*∗*^) in the system.

The equilibrium point can be an ESS, if and only if, it is a both strict Nash equilibrium and a pure strategy Nash equilibrium [61]. Thus, *E*_9_(*x*^*∗*^, *y*^*∗*^, *z*^*∗*^) is not an ESS under any conditions, because it is a mixed-strategy equilibrium point. According to Lyapunov's method, this study analyzes the stability of the remaining eight equilibrium points and identifies the condition forming ESS in the waste separation supervision system. The necessary and sufficient condition for the system that evolves to an ESS is that all the eigenvalues of the Jacobian matrix is not-positive [15]. We obtained the Jacobian matrix through deriving the first partial derivative of equation (6), that is,

(7) $$\begin{array}{c} J=\left[\begin{array}{ccc} \left(1-2x\right)\left[y\left(H_{1}+f_{1}\right)+R_{1}-C_{1}\right] & x\left(1-x\right)\left(H_{1}+f_{1}\right) & 0\\ y\left(1-y\right)\left[-z\left(1-a\right)f_{2}-H_{1}-f_{1}-af_{2}\right] & m & y\left(1-y\right)\left(1-x\right)\left(1-a\right)f_{2}\\ z\left(1-z\right)\left(y-1\right)f_{2}\left(1-a\right) & z\left(1-z\right)\left(x-1\right)f_{2}\left(1-a\right) & \left(1-2z\right)\left[\left(xy-x-y+1\right)f_{2}\left(1-a\right)-C_{3}\right] \end{array}\right]\text{,} \end{array}$$

where *m* equals to (1 − 2*y*)[(1 − *x*)*z*(1 − *a*)*f*_2_ − *x*(*H*_1_+*f*_1_+*af*_2_)+*f*_1_+*H*_2_ − *C*_2_+*af*_2_].

The eigenvalues of each equilibrium point (eight pure strategy solutions) are obtained by bringing these points into the Jacobian matrix. The eigenvalues of equilibrium point are shown in Tables 2, and 3 lists the corresponding stability conditions of the system.

As shown in Table 3, *E*_1_(0, 0, 0), *E*_2_(0, 0, 1), *E*_3_(0, 1, 0), *E*_5_(1, 0, 0), *E*_7_(1, 1, 0) can be the ESS in the waste separation supervision system. When *R*_1_ < *C*_1_, *af*_2_ < *C*_2_ − (*f*_1_ + *H*_2_) and *f*_2_ − *C*_3_ < *af*_2_ (i.e., condition ①), the eigenvalues corresponding to *E*_1_(0, 0, 0) meet the requirements for ESS. In this case, the stability strategy of three participants is {non-classification behavior, negative participation management, loose supervision}. The first inequality *R*_1_ < *C*_1_ shows that when the revenue for residents from waste separation is less than cost, residents would choose non-classification behavior. From the second inequality *af*_2_ < *C*_2_ − (*f*_1_ + *H*_2_), it is found that when the penalty for property service enterprises is less than the difference between the cost of positive participation management and total benefits, property service enterprises would choose negative participation management. According to the third inequality *f*_2_ − *C*_3_ < *af*_2_, when the difference between the fines received by the government under strict supervision and the additional regulatory costs is less than the fines received under loose supervision, the government would choose loose supervision. When the previousconditions are satisfied, the results show that the mandatory waste separation policy is not effectively implemented because property service companies fail to play a regulatory role, and residents do not separate waste in the daily lives.

When *R*_1_ < *C*_1_, *f*_2_ < *C*_2_ − (*f*_1_ + *H*_2_) and *f*_2_ − *C*_3_ > *af*_2_ (i.e., condition ②), the eigenvalues corresponding to *E*_2_(0,0,1) are all less than zero. The first inequalities in condition ② are the same as those in condition ①. The second inequality *f*_2_ < *C*_2_ − (*f*_1_ + *H*_2_) shows that when the penalty for property service enterprises is less than the difference between the cost of positive participation management and total benefits, property service enterprises would choose negative participation management. The third inequality *f*_2_ − *C*_3_ > *af*_2_ means that when the difference between the fines received by the government under strict supervision and the additional regulatory cost exceeds the fines received under loose supervision, the government would choose strict supervision. At equilibrium point *E*_2_(0,0,1), the corresponding stable strategy is {non-classification behavior, negative participation management, strict supervision}.

When *f*_1_ < *C*_1_ − (*H*_1_ + *R*_1_) and *af*_2_ > *C*_2_ − (*f*_1_ + *H*_2_) (i.e., condition ③), the corresponding stability strategy of three participants is {non-classification behavior, positive participation management, loose supervision}. The first inequality *f*_1_ < *C*_1_ − (*H*_1_ + *R*_1_) shows that when the penalty for residents is less than the difference between the cost of separating waste and total benefits, residents would choose non-classification behavior. From the second inequality *af*_2_ > *C*_2_ − (*f*_1_ + *H*_2_), it is found that when the penalty for property service enterprises exceeds the difference between the cost of positive participation management and total benefits, property service enterprises would passively participate in waste separation management.

When *R*_1_ > *C*_1_ and *H*_2_ < *C*_2_+*H*_1_ (i.e., condition ④), the stability strategy of three participants is {classification behavior, negative participation management, loose supervision}. The first inequality *R*_1_ > *C*_1_ shows that when the revenue for residents from waste separation exceeds separation cost, residents would choose classification behavior. From the second inequality *H*_2_ < *C*_2_+*H*_1_, it is found that when the subsidy to property service enterprises is less than the total cost of positive participation management (including investment cost and reward for residents), property service enterprises would choose negative participation management. When the previous conditions are satisfied, the results of the tripartite evolutionary game model suggest that residents will sort their waste only if the benefits of sorting exceed the costs in the absence of any incentives and penalties.

When *f*_1_ > *C*_1_ − (*H*_1_+*R*_1_) and *H*_2_ > *C*_2_+*H*_1_ (i.e., condition ⑤), the stability strategy of three participants is {classification behavior, positive participation management, loose supervision}. The first inequality *f*_1_ > *C*_1_ − (*H*_1_+*R*_1_) shows that when the penalty for residents exceeds the difference between the cost of separating waste and total benefits, residents would choose classification behavior. From the second inequality *H*_2_ > *C*_2_+*H*_1_, it is found that when the subsidy to property service enterprises is higher than the total cost of positive participation management, property service enterprises would choose positive participation management. When the previous conditions are achieved, the mandatory waste separation policy can be effectively implemented, representing that the waste separation regulation system can evolve to the optimal stable strategy. In other words, the government entrusts properties to supervise the waste separation supervision, and residents separate waste in their daily life.

## 4. Numerical Simulation

Numerical simulations were performed using Matlab R2018a software to show the behavioral strategies of residents, property service enterprises, and government and the main influencing factors of the evolution path in the waste separation supervision system. First, this paper simulates the effects of three participants' initial intentions on the evolutionary process under condition ⑤ (ESS is unique and is *E*_7_(1, 1, 0)). Then, this study simulates the influence of reward, subsidy, and punishment on system evolution.

There are the following reasons for numerical simulation with *E*_7_(1, 1, 0) as an example: Studies on municipal solid waste management demonstrated that government-led governance does not work, requiring multiagent collaborative participation governance [62, 63]. The government assigns environmental responsibility to citizens and companies, which is regarded as an effective approach to governance [64]. Meanwhile, the practical experience in waste management suggested that Chinese government pays attention to encourage the residents and companies to engage in waste management and appropriately decentralize power [65]. Furthermore, related studies proved that the government will gradually decrease intervention under a mature waste recycling industry [66]. From the view of theoretical studies and practical experience, *E*_7_(1, 1, 0) is an optimal and realistic ESS. Thus, this paper simulated the influence of initial intention, reward, subsidy, and punishment on system evolution using *E*_7_(1, 1, 0) as an example.

In order not to lose the generality, this study supposed that the values of all parameters are greater than zero. We refer to the study of Luo and Zhao [54] and set the values of parameters as follows: *C*_1_=3, *R*_1_=2, *f*_1_=1, *C*_2_=6, *H*_1_=2, *H*_2_=10, *f*_2_=10, *C*_3_=4, *a*=0.7.

### 4.1. Initial Intention

In this study, the following three scenarios were set to analyze the impact of three participants' initial intention on evolution path in the system. The results are illustrated in Figure 2.

1. Scenarios (a) is {*x*_0_, *y*_0_, *z*_0_*|x*_0_ ∈ (0.2, 0.5, 0.8), *y*_0_=0.5, *z*_0_=0.5} (see Figure 2(a)).
2. Scenarios (b) is {*x*_0_, *y*_0_, *z*_0_*|y*_0_ ∈ (0.2, 0.5, 0.8), *x*_0_=0.5, *z*_0_=0.5} (see Figure 2(b)).
3. Scenarios (c) is {*x*_0_, *y*_0_, *z*_0_*|z*_0_ ∈ (0.2, 0.5, 0.8), *x*_0_=0.5, *y*_0_=0.5} (see Figure 2(c)).

In the previous three scenarios, the evolution paths of residents, property service enterprises, and governments are represented by the black lines, red lines, and blue lines in Figure 2, respectively. As presented in Figure 2, the system finally converges to *E*_7_(1, 1, 0) under different initial strategies. The evolution speed of property service enterprises choosing positive participation management slows down slightly with the increase of *x*_0_ value (see red lines in Figure 2(a)). When the value of *z*_0_ level increases, the government slowly evolves into loose supervision (see blue lines in Figure 2(c)). However, the speeds for three participants evolved into the stability strategy *E*_7_(1, 1, 0) are gradually increased with an increasing value of *y*_0_ (see Figure 2(b)). This indicated that the active participation of property service companies is crucial to residents' behavior supervision.

### 4.2. Reward

To analyze the impact of reward on evolution path and speeds of three participants, we set *H*_1_ = 2 as the base value and performed sensitivity analysis applying the way of −50% and +50%. The initial intentions are taken as *x*_0_ = 0.5, *y*_0_ = 0.5, *z*_0_ = 0.5. The rewards to residents are 1 (−50%), 2, 3 (+50%). The evolutionary paths of the three participants are illustrated in Figure 3.

We can see from Figure 3 that the change in reward *H*_1_ influences the evolutionary path of the system to the stable strategies. The black lines in Figure 3 show the evolution path of residents, red lines show the evolution path of property service enterprises, and blue lines show the evolution path of governments, and the level of rewards to residents can been seen in the legend. The higher the reward to residents, the faster the evolution speed of residents to classification behavior (see black lines in Figure 3). The evolution speed of property service enterprises into the stable strategy of positive participation management is negatively related to the reward for residents (see red lines in Figure 3). The evolutionary paths of the government basically overlap under scenarios of the low, middle, and high levels of reward *H*_1_ (see blue lines in Figure 3). It means that the government's behavior strategy is not affected by the reward to residents.

### 4.3. Subsidy

We set the value of subsidy *H*_2_ for property service enterprises as 5 (−50%), 10, and 15 (+50%) and observed the evolution path of three participants. The results are presented in Figure 4.

Figure 4 illustrates the evolution path of three participants at different subsidy levels. The black lines, red lines, and blue lines are the evolution paths of residents, property service enterprises, and governments, respectively. The speed of property service enterprise evolves into positive participation management more quickly at high subsidy levels than medium subsidy levels. However, when the subsidy *H*_2_ is low (*H*_2_=5), residents and property service enterprises will not evolve to the stable strategy. As shown in Figure 4, the government eventually tends to the stable strategy of loose supervision at the three subsidy levels. This suggests that the increasing subsidy to property service enterprises has little influence on the behavioral decision-making of government.

### 4.4. Penalty

We set high, medium, and low levels of penalty and observe changes in the system evolution. The penalties for residents are 0.5 (−50%), 1, and 1.5 (+50%), that is, *f*_1_={0.5, 1, 1.5}. The penalties for property service enterprises are 5 (−50%), 10, and 15 (+50%), that is, *f*_2_={5, 10, 15}. The evolutionary paths of the system are shown in Figure 5.

Figure 5(a) illustrates the evolution path of the three participants when the penalty for resident changes.  Figure 5(b) illustrates the evolution path of the three participants when the penalty for property service enterprise changes. The black lines, red lines, and blue lines indicate the evolution paths of residents, property service enterprises, and governments, respectively. The specific values of penalties are shown in the legend. The higher the penalty for residents, the faster the evolution speed of residents to classification behavior (see black lines in Figure 5(a)). With the change of penalty for residents, the evolution path of property service companies and the government almost coincides. This indicates that an increase in penalties for non-classification enhances the evolution speed of residents to the optimal stabilization strategy, while having no significant effect on the evolution speed of property service companies and the government.

With the increase of the penalty for property service enterprise, the evolution speed of residents (see black lines in Figure 5(b)) and the property service enterprises (see red lines in Figure 5(b)) accelerates, while that of the government slows down slightly (see blue lines in Figure 5(b)). This means that increasing the penalty for property service enterprises not only promotes participation of property service enterprises in waste separation management but also improves waste separation behavior of residents.

## 5. Discussion

According to the solution of the tripartite evolutionary game model, it can be concluded that when the mandatory waste separation policy is not implemented, the residents will separate waste if the benefit gained from waste separation is greater than the cost of classification. After the implementation of mandatory waste separation, there exists the rewards and penalties and the supervision of waste separation inspectors. Residents will participate in waste separation when the penalty for them is greater than the difference between the cost and benefit of separation. The evolutionary game model of supervision mechanism can achieve the optimal stability strategy (i.e., {Classification behavior, Positive participation management, Loose supervision}) when the following conditions are satisfied: (1) the penalty for resident who do not separate their waste is higher than the difference between classification cost and the total benefit of classification; (2) the subsidy to property services enterprise is greater than the total cost of positive participation management. The result is similar with Chen and Gao [59] who used multi-agent-based simulation to investigate the learning measures of residents' waste separation behavior. This finding also echoes the study of Zhang et al. [58] who found that higher waste separation benefits and lower costs can increase residents' participation rates of waste separation. This indicated that it is necessary not only to reduce the cost of sorting waste and increase the penalty for non-classification but also to reduce the management costs of property service companies, as well as to increase subsidies for them.

The results of numerical simulation indicated that under the two conditions that satisfy the optimal stabilization strategy, residents will still adopt the strategy of classification behavior after the government tends to the loose supervision. This finding echoes the result of Yang et al. [65]. The possible reason is that residents were compelled to conduct waste separation at the beginning of the mandatory policy. After some time, waste classification behavior became a daily habit for residents and internalized into a social norm [66]. Therefore, even if the government adopts loose supervision, residents will still choose classification behavior. Property service enterprises were compelled to engage in waste separation management in the community under the supervision of the government. Corporate social responsibility is positively related to revenue [67]. The intention of property service enterprises to participate in waste separation management is increasing with the increasing revenue. Thus, in the case of lax government supervision, property service enterprises still choose the strategy of positive participation management.

Interestingly, residents evolved slower to a stability strategy than property service enterprises. The main reason for this phenomenon is that the cost of performing waste separation exceeds the rewards for residents. Residents are more sensitive to cost and losses than benefits [68], so they are reluctant to sort their waste when the perceived cost is higher than reward [69, 70]. However, residents will gradually and slowly evolve into classification behavior under the impact of social norms [71]. Compared with residents, property service enterprises are more rational and pursue the maximization of profits. After balancing the cost and benefit, property service enterprises will quickly adapt their decision-making and evolve faster to a stable strategy than residents.

The simulation results of the sensitivity analysis showed that initial intention, rewards, subsidies, and penalties influence the evolutionary path of the system.

First, the higher the intention of property service enterprises to actively participate in management, the faster the evolution of three stakeholders into the stable strategy. The finding may be caused by the reason that property service enterprises play a role in connecting the relationship between residents and the government. With the increased participation of property service enterprises, reward and penalty measures for residents can be effectively implemented. Residents will choose classification behavior to avoid penalty or get reward [72], thus they quickly evolve into classification behavior when property service enterprises' intention to actively participate in management increases. When property service enterprises actively participate in waste separation management, the pressure on government can be relieved. The government quickly evolves to the stable strategy of loose supervision. Therefore, increasing the willingness of the property service enterprise to participate in management is conducive to the supervision system evolution to optimal stability strategy.

Second, the higher the reward for residents, the more likely residents tended to sort waste. The result is in line with the finding of Duan et al. [73] who found that increasing rewards for non-polluting behavior can facilitate the evolution of stakeholders towards the stable state. Meanwhile, an increase in reward for resident implies that the management cost increases, and property service companies are less motivated to participate in waste separation management. With the increasing reward to residents, the evolution speed of property service enterprises into positive participation management is decreasing. As a promoter and supervisor of waste separation management, the government will consider social and ecological benefits and take measures to motivate enterprises to participate in waste separation management [65]. Therefore, property service enterprises will ultimately evolve to the stable strategy of positive participation management. As the participation of property service enterprises improves, the government will progressively decrease the regulation and evolve to the stability strategy of loose supervision.

Third, the higher the subsidy, the more willing property service companies would actively participate in waste separation supervision. This finding agrees with the result of Wang et al. [74]. The reason may be that the property service enterprise can get stable revenue when they positively participate in waste separation management. Property service enterprises can receive government subsidies and perform their corporate social responsibilities, which effectively reduces the occurrence of speculation behavior. However, when the subsidy is low, property service enterprises are reluctant to participate in waste separation management because revenue is lower than cost. The conclusion is similar to the study of Mak et al. [75] who found that enterprises are reluctant to invest in waste separation if the associated cost is too high. Due to the negative participation of property service enterprises, the residents who separate waste cannot get the rewards, and their revenue is reduced. Then, the probability of residents adopting classification behavior decreases.

Fourth, the higher the penalty for non-classification behavior, the faster residents and property service enterprises evolve to the optimal stabilization strategy. This is similar to the results of Zhang [57]. The reason could be that residents restrict their behaviors to avoid risks (i.e., fines) and prefer to choose classification behavior. The penalty for resident become a part of the property service enterprise's revenue, and an increase in the penalty for resident means that the property service enterprise's revenue increases. Therefore, property service enterprises prefer to choose positive participation management when the penalty for resident increases. The government is less sensitive to the penalty for residents. This finding agrees with the result of Wu et al. [17] and is confirmed in reality. Penalty measures have been promoted in some cities where waste separation is mandatory, such as Beijing, Shanghai, and Shenzhen, and fines for residents refusing to separate waste vary. For example, the fine in Beijing and Shanghai for residents who fail to sort their waste is between 50 yuan and 200 yuan (about US$7.91–31.66), and Xiamen and Shenzhen fine up to 1000 yuan (about US$ 157.12) [76]. In addition, the penalty for property service enterprises not only promotes participation of property service enterprises in waste separation management but also improves residents' waste separation behavior. The possible reason is that with the penalty for property service enterprise increases, the actual input cost of property service enterprise also increases. To maximize revenue or avoid penalties, property service enterprises' enthusiasm for participating in waste separation management increases [73]. Therefore, property service enterprises evolve rapidly to the stable strategy of positive participation management. With the participation of property service enterprises, residents who do not sort waste are more likely to be penalized. As a result, residents quickly evolve into the stable strategy of classification behavior. However, the increase in the penalty for property service enterprises means that the government needs to strengthen supervision. Therefore, the evolution speed of the government into the strategy of loose supervision slightly decreases when the penalties for property services enterprise increase.

## 6. Conclusions and Policy Recommendations

This paper structured a tripartite evolutionary game model for the waste separation supervision system to analyze the behavioral decision-making of residents, property service enterprises, and the government and explored the influence of the main parameters on the ideal stable strategy of the system through numerical simulation analysis. The following conclusions are received: (1) Without regulation, only when the benefits of classification outweigh classification costs, will residents participate in waste separation. (2) Under the supervision of government and property service companies, the regulatory mechanism of waste separation will reach the optimal stable strategy when the following conditions are satisfied: ① the penalty for non-classification is higher than the difference between classification cost and the total benefit of classification; ② the subsidy to property services enterprise is greater than the total cost of positive participation management. (3) Compared with improving the residents' initial intention to separate waste, improving the willingness of property service enterprises to actively participate in waste separation management is more conducive to the evolution of three stakeholders into the ideal stable state. (4) The reward and penalty have positive impacts on the evolution path of residents into classification behavior. When the reward and penalty increased, the residents quickly evolved to the stable strategy of classification behavior. (5) The subsidy and penalty positively affect the evolution path of property service enterprise into positive participation management, and property service enterprise is more sensitive to subsidy than penalty. When subsidy is low, the waste separation supervision system will not evolve to the ideal stable state.

Based on the previous conclusions, we put forward some policy recommendations to establish an effective supervision mechanism and promote residents to conduct waste separation practices.

1. The important role of the property service enterprise should be valued when calling on residents to actively participate in the practice of waste separation. The government should delegate the power of supervision to property service enterprises, enabling them to give full play to the autonomy of grassroots organizations and residents. The government should strengthen the incentive system to effectively encourage property service enterprises to actively engage in the management of household waste separation. Training for waste separation supervisors may be an effective way to reduce the management costs of property service companies. Property service companies can regularly train waste separation instructors on how to spread relevant knowledge to residents and how to effectively persuade and supervise the behavior of nonclassification, thus reducing labor costs. The government can provide special financial subsidies, tax concessions, and preferential policies to property service enterprises. At the same time, a variety of penalties can be applied to avoid the speculative behavior of property service enterprises, such as double fines, credit score deductions, and forced closure.
2. The government should strengthen waste separation propaganda to increase residents' willingness to separate waste. Publicity channels, such as posters, TV commercials, and short video platforms, can be widely used to disseminate the standards, knowledge, and skills of waste separation for the public. The government should also train waste separation instructors to improve their communication skills to discourage non-separation behavior. A public poll should be conducted to understand what management measures are acceptable to residents before implementing regulation. In addition, training residents on waste separation skills is also an effective way to reduce the cost of separating waste. Delicacy management of waste separation supervision needs to be urgently strengthened. First, the government should build a big data supervision platform and utilize intelligent technology to implement waste separation supervision. Second, an evaluation system for domestic waste separation should be established to ensure that property service companies seriously carry out waste management. Third, in order to achieve supervision between residents and property service companies, the government should provide a complaint hotline for residents. Residents can report property service companies to government departments if they violate the rules or fail to act.
3. More detailed incentives and penalties for residents should be announced at the community level to motivate residents to carry out waste separation practices. Property service companies should take a series of measures to motivate residents to form the habit of waste separation. They could install smart waste bins that give residents economic rewards according to their credit points earned from waste separation and regularly organize activities for residents to exchange their points for gifts. Management rules based on the resident characteristics should be formulated, for example, the opinion survey could be conducted to understand reward measures that residents prefer. Before residents form the habit of separating waste, the penalty for nonseparation behavior can be increased to improve residents' speculative costs and perception of deterrence. By using technical means such as the installation of monitoring and code traceability, the behavior of residents can be fully regulated to prevent non-compliance. Property service companies can take a wide range of penalties, such as garbage fees and fines. A list of penalty outcomes could be posted in the community to remind residents that regulation exists and is effective.

The present study confirms the feasibility of property service companies to regulate residents' waste separation behavior and provides new ideas for waste separation management in China and other developing countries. The study still includes certain limitations, which can be addressed in further works. First, we mainly studied the behavior strategies of residents, property service enterprises, and governments under the waste separation supervision system. Future research could introduce other stakeholders into the game model of waste separation supervision to analyze the interaction among multi-agent, such as the interaction between residents and non-governmental organizations, and the interaction between residents and neighborhood committees. Second, this study has conducted only the numerical simulation analysis to verify the feasibility of the waste separation supervision system. In the subsequent study, real data can be collected through field trials or case studies to verify the replicability of the waste separation supervision mechanism considering tripartite participation.

## Figures and Tables

**Figure 1:** The tripartite game tree.

**Figure 2:** The impact of initial intention on system evolution. (a) The impact of residents' initial intention on system evolution. (b) The impact of property service enterprises' initial intention on system evolution. (c) The impact of governments' initial intention on system evolution.

**Figure 3:** The impact of reward on system evolution.

**Figure 4:** The impact of subsidy on the system evolution.

**Figure 5:** The impact of penalty on system evolution. (a) The impact of penalty for resident on system evolution. (b) The impact of penalty for property service enterprise on system evolution.

**Table 1:** The payoff matrix.

Resident	Property service enterprise			
	Positive participation management (*y*)		Negative participation management (1 − *y*)	
	Government		Government	
	Strict supervision (*z*)	Loose supervision (1 − *z*)	Strict supervision (*z*)	Loose supervision (1 − *z*)
Classification behavior (*x*)	*R*_1_+*H*_1_ − *C*_1_	*R*_1_+*H*_1_ − *C*_1_	*R*_1_ − *C*_1_	*R*_1_ − *C*_1_
	*R*_2_+*H*_2_ − *C*_2_ − *H*_1_	*R*_2_+*H*_2_ − *C*_2_ − *H*_1_	*R*_2_	*R*_2_
	*R*_3_ − *C*_3_ − *H*_2_	*R*_3_ − *H*_2_	*R*_3_ − *C*_3_	*R*_3_

Non-classification behavior (1 − *x*)	−*f*_1_	−*f*_1_	0	0
	*f*_1_+*H*_2_ − *C*_2_	*f*_1_+*H*_2_ − *C*_2_	−*f*_2_	−*af*_2_
	*R*_3_ − *C*_3_ − *H*_2_	*R*_3_ − *H*_2_	*f*_2_ − *C*_3_ − *C*_4_	*af*_2_ − *C*_4_

**Table 2:** The eigenvalues of equilibrium point.

Equilibrium point	Eigenvalues			Evolutionary stability
	*λ*_1_	*λ*_2_	*λ*_3_	
*E*_1_(0, 0, 0)	*R*_1_ − *C*_1_	*f*_1_+*af*_2_+*H*_2_	*f*_2_(1 − *a*) − *C*_3_	Condition①
*E*_2_(0, 0, 1)	*R*_1_ − *C*_1_	*f*_1_+*f*_2_+*H*_2_ − *C*_2_	*C*_3_ − *f*_2_(1 − *a*)	Condition②
*E*_3_(0, 1, 0)	*H*_1_+*f*_1_+*R*_1_ − *C*_1_	*C*_2_ − *f*_1_ − *af*_2_	−*C*_3_	Condition③
*E*_4_(0, 1, 1)	*H*_1_+*f*_1_+*R*_1_ − *C*_1_	*C*_2_ − *f*_1_ − *f*_2_ − *H*_2_	*C*_3_	Unstable
*E*_5_(1, 0, 0)	*C*_1_ − *R*_1_	*H*_2_ − *H*_1_ − *C*_2_	−*C*_3_	Condition④
*E*_6_(1, 0, 1)	*C*_1_ − *R*_1_	*H*_2_ − *H*_1_ − *C*_2_	*C*_3_	Unstable
*E*_7_(1, 1, 0)	*C*_1_ − *H*_1_ − *f*_1_ − *R*_1_	*H*_1_+*C*_2_ − *H*_2_	−*C*_3_	Condition⑤
*E*_8_(1, 1, 1)	*C*_1_ − *H*_1_ − *f*_1_ − *R*_1_	*H*_1_+*C*_2_ − *H*_2_	*C*_3_	Unstable

**Table 3:** Equilibrium stability conditions of the system.

Equilibrium point	Stability condition	Number
*E*_1_(0, 0, 0)	*R*_1_ < *C*_1_, *af*_2_ < *C*_2_ − (*f*_1_+*H*_2_), *f*_2_ − *C*_3_ < *af*_2_	①
*E*_2_(0, 0, 1)	*R*_1_ < *C*_1_, *f*_2_ < *C*_2_ − (*f*_1_+*H*_2_), *f*_2_ − *C*_3_ > *af*_2_	②
*E*_3_(0, 1, 0)	*f*_1_ < *C*_1_ − (*H*_1_+*R*_1_), *af*_2_ > *C*_2_ − (*f*_1_+*H*_2_)	③
*E*_5_(1, 0, 0)	*R*_1_ > *C*_1_, *H*_2_ < *C*_2_+*H*_1_	④
*E*_7_(1, 1, 0)	*f*_1_ > *C*_1_ − (*H*_1_+*R*_1_), *H*_2_ > *C*_2_+*H*_1_	⑤

## Data Availability

The datasets used and analyzed during the current study are available from the corresponding author on reasonable request.
